# Development of Radiofrequency Ablation Generator and Balloon-Based Catheter for Microendoluminal Thin-Layer Ablation Therapy Using the Rat Duodenum as a Model of Low-Impedance Tissue

**DOI:** 10.1155/2021/9986874

**Published:** 2021-09-23

**Authors:** Jana Nociarova, Marek Novak, Jan Polak, Jan Hrudka, Stefan Porubsky, Michal Koc, Jozef Rosina, Aleksandr N. Grebenyuk, Radek Sery, Robert Gurlich, Jan Hajer

**Affiliations:** ^1^Department of Internal Medicine, Third Faculty of Medicine, Charles University, University Hospital Kralovske Vinohrady, Prague 100 34, Czech Republic; ^2^Department of Medical Biophysics and Medical Informatics, Third Faculty of Medicine, Charles University, Prague 100 00, Czech Republic; ^3^Department of Pathophysiology, Third Faculty of Medicine, Charles University, Prague 100 00, Czech Republic; ^4^Department of Pathology, Third Faculty of Medicine, Charles University, University Hospital Kralovske Vinohrady, Prague 100 34, Czech Republic; ^5^Institute of Pathology, University Medical Center of the Johannes Gutenberg University in Mainz, Mainz 55 131, Germany; ^6^Department of Health Protection and Disaster Medicine, Pavlov First State Medical University of St. Petersburg, St. Petersburg 197 022, Russia; ^7^Centre of Toxicology and Health Safety, National Institute of Public Health, Prague 100 00, Czech Republic; ^8^Department of General Surgery, Third Faculty of Medicine, Charles University, University Hospital Kralovske Vinohrady, Prague 100 34, Czech Republic

## Abstract

Radiofrequency ablation (RFA) is a routinely used, safe, and effective method for the tissue destruction. Often, in case of its application in malignant conditions, the extent of tissue destruction is insufficient due to the size of the target lesion, as well as due to the risk of heat-induced damage to the surrounding organs. Nevertheless, there are conditions requiring superficial precise-depth ablation with preservation of deeper layers. These are represented, for example, by mucosal resurfacing in case of Barrett's esophagus or treatment of recurrent mucosal bleeding in case of chronic radiation proctitis. Recently, new indications for intraluminal RFA use emerged, especially in the pancreatobiliary tract. In the case of intraductal use of RFA (e.g., biliary and pancreatic tract), there are currently available rigid and needle tip catheters. An expandable balloon-based RFA catheter suitable for use in such small-diameter tubular organs could be of benefit due to possible increase of contact between the probe and the target tissue; however, to prevent excessive tissue damage, a compatible generator suitable for low-impedance catheter/tissue is essential. This project aimed to develop a radiofrequency ablation generator and bipolar balloon-based catheter optimized for the application in the conditions of low-impedance tissue and (micro)endoluminal environment. Subsequent evaluation of biological effect in vivo was performed using duodenal mucosa in Wistar rat representing conditions of endoluminal radiofrequency ablation of low-impedance tissue. Experiments confirming the safety and feasibility of RFA with our prototype devices were conducted.

## 1. Introduction

Radiofrequency ablation (RFA) is a well-established method for local tissue destruction. It is a treatment modality broadly used for various medical conditions, predominantly as adjuvant therapy for malignancies of solid organs (liver and kidney) [1] and therapy of atrial fibrillation in cardiology [2]. It can be applied via the open, laparoscopic, percutaneous, or endoscopic route [3–5], most recently also using a EUS- (endoscopic ultrasound-) guided RFA probe [6, 7].

The main limitation of the RFA is the insufficient size of destruction that can be produced in large volume lesions. RFA induces desiccation of tissue resulting in coagulative necrosis and, due to the rise in impedance of necrotic tissue, the current stops flowing, which limits the area successfully treated. Another cause of incomplete ablation is the heat-sink effect (defined as local tissue cooling due to the proximity of vessels), preventing the effective temperature from being attained [1, 8].

Contrary to situations, where the depth of ablation is insufficient, several conditions are requiring specifically superficial ablation, for example, benign mucosal conditions (e.g., postradiation proctitis and gastric antral vascular ectasia) [9] and Barrett´s esophagus, representing a common indication for RFA mucosal resurfacing (MR). Mucosal resurfacing involves the physical removal of superficial abnormal tissue followed by regrowth and restoration of normal tissue through a stem cell-mediated healing response [10]. Currently, the most common application of MR is the endoscopic treatment of Barrett's esophagus, a precancerous condition, in which the normal squamous epithelium of the distal esophagus transforms to columnar-lined intestinal metaplasia. In this case, destruction of the mucosa by MR is subsequently followed by restoration of the squamous epithelium [10].

Another possible application of mucosal resurfacing, also most anatomically analogous to MR used for Barrett´s esophagus, is duodenal mucosal resurfacing (DMR). DMR is an innovative endoscopic method for superficial tissue destruction using hydrothermal ablation of proximal duodenum leading to modification of duodenal metabolic and endocrine signaling. According to recently published pilot data, DMR seems to be a promising treatment modality for T2DM (type 2 diabetes mellitus), although further studies are necessary to better understand the underlying mechanisms of the procedure [11–13]. RFA as a method for MR is known to be safe and effective in Barrett´s esophagus. However, it has not been used for DMR so far.

Currently, there are several devices available for endoluminal RFA. In terms of design, they are either inflatable balloon catheters or rigid needle-tip probes. Inflatable balloon catheters aimed at mucosal resurfacing are routinely available only in larger sizes. Rigid catheters are used either transcutaneously or endoscopically, mostly as a method of palliative tumor debulking [14]. Recently, there emerged researches of new smaller diameter inflatable RFA probes specified for intrabiliary use. According to available data, those are designed for deeper tissue ablation rather than mucosal resurfacing as they employ water-filled balloons [15], which have very long ramp-up and ramp-down temperature periods due to the specific thermal capacity of the water resulting in excessive local heat.

The present paper was focused on the balloon-based bipolar radiofrequency catheter and RFA generator development, followed by an evaluation of its effect in microendoluminal environment and low-impedance tissue represented by duodenal mucosa of the Wistar rat.

## 2. Material and Methods

To achieve the goals of this research, a series of experiments followed by custom development of electrical and mechanical instruments were performed before the actual animal experiments. Thus, this section first describes the development of the methodology and instrumentation, and the methodology of animal experiments follows.

### 2.1. Initial Experiments with Commercial Off-the-Shelf Instruments

The first experiments were performed using a commercially available RFA generator (Rita Model 1500X, Angiodynamics) and endoluminal catheter (Habib EndoHPB, EMcision, Ltd. London, UK), which seemed to be the most appropriate instrument in the conditions of our test due to its diameter (8 F = 2,6 mm). Before the animal procedure, the catheter was tested using ex vivo poultry liver and the extent of energies planned to use in the rat duodenum was established. These energies were then applied to the proximal small intestine of the rat, gradually increasing from low to higher energies to avoid unwanted heat-induced damage to the adjacent tissue. Nevertheless, the required histological effect (uniform destruction of superficial mucosa) was not attained (Figure 1(a)). One of the possible causes of this failure was presumed inadequate contact between the catheter and duodenal wall because of the rigid structure of the catheter, while the shape of the duodenum was irregular.

### 2.2. Catheter Development

Based on this observation, we have decided to design our custom-made balloon-based RFA bipolar catheter (Figure 2). The balloon-based catheter is inflated in the place of required ablation and therefore the optimal contact between the RFA probe and target tissue should be ensured. A commercially available balloon catheter (Mustang, Boston Scientific) with custom electrodes manufactured as a flexible printed circuit board—Kapton substrate with electroless nickel gold surface finish copper electrodes)—was designed and manufactured. The length of the electrode was 20 mm. The neighboring conductive traces have opposite polarity, the width of the conductors was 0.3 mm and the spacing between conductors was 0.2 mm. The Kapton substrate with metal electrodes was then glued onto an inflated catheter balloon using flexible B-7000 glue and let harden in the inflated state with partially shrunk PVC tubing over the whole assembly to provide sufficient pressure to the contact region and to prevent unrolling of the Kapton electrode. The high power ablation waveform is applied to the electrodes with a 0.5 mm diameter microcoaxial cable with a length of about 50 cm. This cable is soldered to the gold-Kapton electrode on one side and a 5.5/2.5 mm power connector on the other side.

To further verify the ability of this catheter to cause fully circular ablation, we performed an ex vivo experiment with the use of poultry liver. Using this balloon catheter connected to RFA generator (Effect 8, VIO 300D; ERBE Elektromedizin GmbH, Tübingen, Germany), we achieved a circular effect over the whole length of the electrode (Figure 3(b)), unlike the discontinuous effect of the commercially available rigid probe (Figure 3(a)). Voltage and current to the electrode during ablation were measured using a UNI-T UTD2025C oscilloscope with ×10 probes and a 1 Ohm shunt resistor to measure the current. The voltage and current probes were placed between the unit and electrode. The electrode was placed inside the tissue and inflated. The maximum measured power delivered to the tissue was only 30 W which is 4 times less than the preset value. Despite the fact that we achieved the circular ablation effect, the unit was unable to deliver the preset power. This resulted in a prolonged period of ablation (3 seconds) and approx. 2 mm depth of ablation, which is too excessive for mucosal resurfacing. To better understand this limitation, impedance measurements of various tissue types were performed. The impedance, using our custom electrode, varied between approx. 4 and 7 Ohms, which is below the minimum of acceptable impedance required by current commercially available generators. The output impedance of the generator is most likely higher than the impedance of the electrode, which means that the majority of RF power generated by the unit is not delivered to the tissue but instead is radiated as heat in the generator and cables.

We further confirmed the inability to perform superficial tissue destruction in conditions of low-impedance tissue such as the duodenal wall of the laboratory rat. The required ablation was not achieved (Figure 1(b)).

## 3. Radiofrequency Generator Development

To solve this issue, we have decided to develop our radiofrequency generator (Figure 4). We have adopted the output RF frequency provided by the VIO 300D generator, 400 kHz frequency sine wave, but we have optimized the generator for very-low-impedance RFA balloons (<10 Ohms).

As the main power supply, a commercially available 24 V power supply capable of delivering up to 12 A of current was chosen. An auxiliary (12 V 2 A and 5 V 1 A) power supply is used for the control and logic part of electronics.

The control is separated among two microcontrollers—one for RFA waveform generation and control and the other for the user interface. The user interface board is placed on the front part of the generator and contains several analog and digital inputs and outputs as well as a 4 × 40 alphanumeric LCD and interface for a matrix keyboard. PIC18F87J10 microcontroller was used to control the display and user interface.

The matrix keyboard is placed on the front panel as well. It contains a separate PIC16F1783 which sends the information about pressed keys and length of the button press via UART link to the PIC18F87J10 microcontroller.

The power circuitry consists of several printed circuit boards. The power H-bridge is driven from a 60 V power line. The output from the main 24 V power supply is converted to 60 V with a step-up converter with Texas Instruments LM5022. The maximum continuous power output is 100 W, but the circuit can deliver a peak output power of over 200 W for several seconds. The heat which is generated in the circuit is dissipated mainly in the MOSFET transistor (equipped with an appropriate heat sink) and coil.

The goal of the development was to offer a universal RFA platform to accompany a large variety of RFA catheter balloons and other electrodes. The range of power delivered to the probe can vary from a fraction of watt to over 100 W. To accomplish this task, instead of traditional digital PWM control, the 80 V output power rail is connected to a digitally controlled step-down converter. The output of this step-down converter is then fed directly to the H-bridge which drives the RFA electrode. The step-down converter is based on Texas Instruments LM5116 high-voltage step-down converter. The output voltage of the converter is controlled by a voltage feedback resistor divider formed by a discrete resistor with a value of 100 kOhm and 256-step digital potentiometer Maxim MAX5483. The principle of operation is based on the fact that the LM5116 is a feedback-controller step-down controller which controls the output voltage based on the voltage at the FB pin of the integrated circuit. The 100 kOhm (represented as R1 for following calculations) and digital potentiometer form a resistor divider which can be expressed by the following equation:

(1) $$\begin{array}{c} V_{FB}=V_{\text{out}}\frac{R_{\text{pot}}}{R_{\text{pot}}+R1}. \end{array}$$

*R*1 has a static value of 100 kOhm, *V*_*FB*_ is the voltage at the FB pin, and *V*_out_ is the output voltage of the step-down converter. The value of *R*_pot_ can be controlled digitally in 256 discrete steps up to 10 kOhm. The single step is approximately 39 Ohms. The value of *R*_pot_ which has to be set to achieve the desired voltage *V*_out_ can then be easily determined from the above-mentioned equation:

(2) $$\begin{array}{c} R_{\text{pot}}=R1\frac{V_{FB}}{V_{\text{out}}-V_{FB}}. \end{array}$$

*V*_*FB*_ for LM5116 is 0.8 V. As an example, if an output voltage of 20 V is desired, the *R*_pot_=4.16 *k* Ohm. This corresponds to the digital value of approximately 0 × 6B (108 in decimal) which is to be programmed to the digital potentiometer.

The output of the digitally controlled step-down converter is then fed directly to the H-bridge comprised of four N-channel MOSFETs. The gate driving circuitry comprises two half-bridge LM5104 bootstrap drivers. The control signals are generated by the FSMC module of the PIC16F1783 microcontroller. Both frequency and duty cycle of the output waveform can be digitally controlled. The output of the half bridge is filtered in a low-impedance LC resonant circuit (used in this particular implementation to enable ablation with low-impedance probes).

One of the advantages of the developed generator is that it can track (and in the future precisely control) the energy delivered to the tissue. This is enabled by current and voltage monitoring at the output of the LC circuit. The voltage monitoring is achieved by a Graetz bridge (the output voltage is in the range of tens of volts so the error caused by rectification is negligible). The output voltage is then passed through an RC filter to obtain an effective value of the voltage and conditioned (divided by a factor of 25 and buffered with an operational amplifier) so it can be outputted to the analog input of the microcontroller for sampling.

The precise measurement of the current is, however, more complicated. After several experiments with low-side and high-side shunt resistors which did not yield satisfactory results (mainly because of the high frequency of 400 kHz which is well above the cut-off frequency of most integrated circuits intended for current shunt sensing), a Murata 7000 current sensing transformer with a ratio of 1 : 100 was chosen. The primary winding of the current sensing transformer is connected in series to the circuit, while the secondary is loaded with a 100-Ohm resistor. The current at the secondary is 100x smaller than that in the primary winding. Thus, the voltage generated on the 100-Ohm resistor can be represented by the following formula:

(3) $$\begin{array}{c} U_{\text{curr}\_\text{out}}=\frac{I}{100}R_{2}, \end{array}$$

where *U*_curr_out_ is the voltage on the *R*_2_ resistor and *I*is the current delivered to the RFA probe. The current can then be determined from the voltage on the resistor using the following formula:

(4) $$\begin{array}{c} I=100\frac{U_{\text{curr}\_\text{out}}}{R_{2}}. \end{array}$$

The output on the secondary side resistor is conditioned similarly to the voltage output and outputted to the analog input of the microcontroller.

The actual power delivered to an electric load is represented by the following formula:

(5) $$\begin{array}{c} P_{\text{act}}=U_{\text{act}}I_{\text{act}}, \end{array}$$

where *P*_act_ is the actual power, *U*_act_ is the actual voltage across the load, and *I*_act_ is the current flowing to the load. The energy delivered over a specified time frame from *t*=*t*_0_ to *t*=*t*_1_ with arbitrary current and voltage across and flowing through the load, respectively, can be calculated using the following formula:

(6) $$\begin{array}{c} E=\int_{t_{0}}^{t_{1}}U\left(t\right)I\left(t\right)\text{d}t, \end{array}$$

where *U*(*t*) is the function which represents the voltage over time and *I*(*t*) is the current over time. In a discrete time (more suitable for a digital sampling system), the formula can be rewritten as follows:

(7) $$\begin{array}{c} E=\sum_{t_{0}}^{t_{1}}U\left[t\right]I\left[t\right]\text{dt}. \end{array}$$

However, direct voltage and current sampling would be very impractical in our prototype RFA system due to large requirements on the sampling rate and computing power. The sampling rate must have been of a magnitude of several MHz to achieve good accuracy.

Thus, a different approach was chosen. This approach exploits the characteristics of RFA signals. First, the signals are harmonic. Thus, the power can be interpreted as follows:

(8) $$\begin{array}{c} E=\int_{t=t_{0}}^{t_{1}}U_{\max}\sin\left(t\right)I_{\max}\sin\left(t+\varphi \right)\text{d}t, \end{array}$$

where *U*_max_ and *I*_max_ are peak values of voltage and current, respectively, and *φ* is the phase shift between voltage and current. Measurements with an oscilloscope confirmed that the character of the load (ablated tissue) is almost purely resistive at this relatively low frequency of 400 kHz. This means that the formula above can be simplified to

(9) $$\begin{array}{c} E=\int_{t=t_{0}}^{t_{1}}U_{\max}\sin\left(t\right)I_{\max}\sin\left(t\right)\text{d}t. \end{array}$$

This can be (concerning the load character and the fact that the changes in the tissue are rather slow as opposed to the 400 kHz ablation waveform) rewritten to an approximate form:

(10) $$\begin{array}{c} E=\int_{t=t_{0}}^{t_{1}}U_{\text{eff}}\left(t\right)I_{\text{eff}}\left(t\right)\text{d}t. \end{array}$$

It can also be written in discrete form:

(11) $$\begin{array}{c} E=\sum_{t_{0}}^{t_{1}}U_{\text{eff}}\left[t\right]I_{\text{eff}}\left[t\right]\text{d}t. \end{array}$$

Hence, simultaneous sampling of the effective value of voltage and current without phase difference determination is sufficient to calculate the energy delivered to the tissue. The values of effective voltage and current are sampled with a frequency of 1 kHz; their product is integrated over time and shown on the display.

The output of the LC circuit is provided directly to the BNC connector on the front panel where the probe connects.

The user interface on the 4 × 40 segment display is used to show the parameters of the RF ablation—on-time, off-time, number of pulses, and voltage settings. On the right side, applied energy is shown. The on-time and off-time settings can be used to precisely control the length of ablation pulses and delay between them. The voltage can be regulated from 12 V to 80 V. The ablation can be activated either with a button or with a foot pedal, allowing full control over the device operation and ablation balloon by one person.

### 3.1. Animals and Procedure

#### 3.1.1. Animals

12-week-old male Wistar rats (Charles River, distributed by Velaz, Prague, Czech Republic) were used in the project. Animals were housed under constant ambient temperature (22 ± 1°C) and humidity in a light-dark cycle of 12 : 12 hours and fed ad libitum standard rat chow with free access to water. All procedures involving animals were approved by the institutional ethical committee (under the identification number: 85/2018).

#### 3.1.2. Procedures

Animals fasted 12 hours preoperatively. General anesthesia was induced and maintained with an isoflurane/O_2_ mixture. The abdomen was opened using a midline laparotomy and a 3 mm incision in the prepyloric part of the stomach was made (Figure 5(a)).

Under direct visualization, a wire-guided balloon catheter was inserted into proximal 2 cm of the duodenum (Figure 5(b)). Once the catheter was properly placed, a balloon was inflated to temporarily flatten the duodenal folds (Figure 5(c), white arrow). Ablation of duodenal mucosa was performed using a custom-made RFA generator (3 pulses, each 750 ms, 80 V, pause between pulses 10 ms). In the initial phase of the project, we performed also a sham operation that included the insertion and inflation of the balloon catheter but without a subsequent application of radiofrequency energies.

In pilot experiments, endoscopic examination of the ablated area was also performed to evaluate the macroscopic acute effect of RFA in vivo using a flexible transnasal endoscope (model ENF-P3, Olympus). The endoscope was inserted through the incision in the prepyloric part of the stomach and using a method of direct endoscopy ablated area was evaluated by the examiner (Figure 6).

At the end of the procedure, the abdomen was closed using continuous suturing (Figure 5(d)). Animals were administered analgesics (buprenorphine 0.05 mg/kg i.m.) at the end of the procedure and every 12 hours for 2 days (in survival animals). The tissue harvested from the proximal small intestine was performed immediately after the procedure, 24 hours after the procedure, or 14 days after the intervention. Throughout the study period, animals were intensively observed to detect any signs of distress, painful reactions, or changes in peroral intake. At the end of the experiment, euthanasia was performed by anesthetics overdose.

#### 3.1.3. Tissue Harvest and Histological Evaluation

Under general anesthesia with an isoflurane/O_2_ mixture, a midline laparotomy was performed to obtain samples from the intervened part of the proximal small intestine. Subsequently, euthanasia was performed by anesthetics overdose. The tissue was fixed overnight in 4% formalin and then samples were orientated and embedded in paraffin blocks. Sections were cut at 4 *μ*m thickness and mounted on glass slides before being stained with hematoxylin and eosin according to the standard procedure [16]. Analyses of histological samples by a board-certified pathologist assessed the extent of tissue ablation. The digital images were obtained with the use of the digital slide scanner (Pannoramic Scan II, 3DHISTECH Ltd., Hungary). When evaluating the degree of thermal injury, the presence of the epithelial layer is assessed. If the epithelial layer is present, the thermocoagulation artifacts are seeked for. In case of successful tissue damage, signs of intravital reaction are noticed—fibrin precipitation, blood clots, and neutrophils. In the case of necrosis, hypereosinophilia and loss of nuclear staining are present.

## 4. Results

### 4.1. Custom Catheter and Generator Development

The construction of a custom catheter for radiofrequency ablation of duodenal mucosa in a rat model was successful with the subsequent verification. The generator is capable of generating RF pulses with varying voltage amplitude and length. Moreover, the generator is optimized for low-impedance balloon catheters and high energy to surface area ratio ablation. Unlike commercially available solutions, the developed generator provides useful debug data like impedance measurement and total delivered energy to the tissue. The technology for hand-manufacturing of custom balloon catheters allows for great flexibility in terms of the diameter of the balloon and length of the ablated portion of the tissue. It was found that Kapton or another high-temperature polymer should be used as the temperature on the surface of the electrodes far exceeds 100°C (the ablation was connected with the immediate generation of steam at the surface of the electrodes). Next, the electrodes should not be reprocessable as the ENIG coating of the copper electrodes tends to degrade and the necrotic tissue forms an isolation layer which is very hard to be cleaned off the electrodes.

### 4.2. In Vivo Assessment of Ablation Effect

Radiofrequency ablation of duodenal mucosa was successfully performed with the designed RFA generator and bipolar balloon-based RFA catheter optimized for use in conditions of low-impedance tissue. The wattage and exposure time was determined based on the previous testing followed by histological evaluation. During the endoscopic examination of the treated area, we observed circular discoloration of mucosa in place, where RF energy was applied, without any immediate signs of hemorrhage, ulcerations, or perforation (Figure 6).

No major procedure-related adverse events were observed. All animals survived without any distressing behavioral patterns.

### 4.3. Histopathological Assessment

Histological examinations determined the presence and the extent of ablation. In the specimens removed directly after application of RFA energy, microscopically the ablated area showed hemorrhagic necrosis of the epithelium and lamina propria mucosae, with the adjacent fibrin coagulum, lamina muscularis mucosae is mostly intact, and there are isolated necrotic smooth-muscle cells present (Figure 7(b)). The extent of tissue damage ranged from partial ablation (Figure 7(b)) to transmural necrosis (Figure 7(c)) depending on delivered energy. In the samples obtained on the 14^th^ day after the procedure, macroscopically there were no signs of duodenal wall perforation or stricture. As demonstrated in Figure 7(d), microscopically the physiological architecture of the epithelium was preserved.

## 5. Discussion

In our study, we developed a prototype of an RFA generator specifically for use in low-impedance tissue aimed at superficial tissue destruction without injury to deeper structures. Our experiments demonstrated promising results with the use of an inflatable balloon-based catheter due to its enhanced contact with the mucosa.

Regarding commonly used RFA of solid organ tumors, the range of ablation is usually limited by the size of the tumor and the rise of the impedance of necrotic tissue in large volume tumors, leading to reduced current flow and insufficient procedure. Yet, there are conditions when RFA is limited not only by the actual size of the target lesion but also by the risk of thermal injury to the adjacent tissue. Such a situation is represented, for example, by the treatment of malignant biliary stenosis or as a cytoreductive palliative measure for unresectable pancreatic tumors, as the pancreas is a highly thermosensitive organ in the proximity of large vessels and intestinal walls. Excessive thermal injury in this area may lead to serious consequences [8, 17]. As regards the use of RFA in the biliary tract, it is also technically challenging to ensure appropriate circumferential contact between the rigid RFA probe and the duct wall (e.g., in case of bile duct dilation, bending of the bile duct, or the nodular appearance of neoplasm) [18]. We believe that a balloon-based catheter would be more advantageous in targeting such lesions, compared to currently available rigid or needle-tip catheters. Balloon catheter should ensure more precise contact between the RFA electrodes and the tissue resulting in more uniform and continuous tissue damage. At the moment, there are several devices available for endoluminal RFA in the gastrointestinal tract. Circumferential balloon catheters are available only in larger sizes, for example, Barrx 360 Express RFA balloon catheter (Medtronic Inc.), a self-adjusting balloon with its outer diameter from 18 mm to 31 mm, and the same size earlier generation Barrx 360 RFA balloon catheter (Medtronic Inc.) without autosizing ability. These are used specifically for the treatment of Barret's esophagus [19, 20]. Several other devices are used for focal mucosal treatment, either as an initial treatment in a more limited area of abnormal mucosa or as a follow-up treatment after initial circumferential treatment (Barrx 60 and 90 focal RFA catheters, Barrx Ultra Long focal RFA catheter, Medtronic Inc.) [14]. Habib Endo HPB catheter (EMcision Ltd.), Habib EUS-RFA catheter (flexible, monopolar, can be inserted through 19- or 22-gauge FNA needle), and ELRA™ (STARmed Co.) are needle-tip probes used for intraductal ablation [14, 21]. Previous clinical experience with biliary RFA treatment appears to be promising, but data regarding its benefit in terms of survival remain conflicting [22–24], mostly because of the small sample size used in studies, heterogeneous etiologies, localization of strictures, and lack of prospective data. The most commonly reported adverse events of biliary RFA are hemobilia, strictures, liver infarction, pancreatitis, and pseudoaneurysm of the hepatic artery [25]. To avoid unintended thermal damage novelty temperature-controlled RFA systems (ELRA™, STARmed Co.) had been studied [26]. These systems automatically shut down when the temperature reaches the preset target and reactivate the energy delivery to maintain the preset temperature. Studies comparing between power-controlled (Habib Endo HPB) and temperature-controlled (ELRA™) are lacking [22]. Nevertheless, all of the above-mentioned platforms use rigid probes or large-size balloon catheters. Routinely used smaller diameter RFA balloon catheters for microendoluminal therapy are not yet available. However, there are emerging new studies focused on the use of intraductal inflatable balloon catheters in animal models. Inoue et al. recently informed about promising results with achieving circumferential even ablation in porcine bile ducts with the use of the inflatable catheter prototype [15]. In this study, reported depths of ablation were 3.46 mm and 5.07 mm, which seem to be promising for the use in malignant biliary obstruction but are still too vast for the use in benign mucosal conditions or mucosal resurfacing methods. The design of catheters is intended rather for deep tissue ablation as it is filled with water during the procedure. This is the primary differentiating factor. Liquid-filled balloons lack the capability of superficial tissue ablation, as opposed to our solution. Unlike the prior art, we present a technical solution for manufacturing high-temperature capable catheters. Based on our experience, the material used for manufacturing currently available catheters disintegrates at a temperature of above 100°C which limits the possible applications. In case of superficial ablation, the goal is to heat and cool down the catheter as quickly as possible to cause the only destruction of the thin layer and leave the deeper layers intact. Thus, the main priority of this project was to develop devices capable of achieving even and precise depth ablation in small-diameter tubular organs. For superficial ablation, high power delivered over a short period is essential. However, the maximum power (measured by the oscilloscope sensing voltage and current) that the commercially available generator combined with our catheter could provide in the experiment was only 30 W. Therefore, we constructed a prototype of an RFA generator with an optimized power stage for low-impedance catheters (up to 15 Ohms). Using this generator with our catheter (with 150 W power), we were finally able to control the extension of circular tissue damage in vivo in an animal model ranging from partial ablation to transmural necrosis, depending on delivered energy. The main possible improvement of the generator design is to enhance the computational capability (by using a microcontroller with higher performance) to be able to precisely measure the delivered energy to the site in real time and cut-off at predefined energy. While the consistency with time and voltage specified dosing of energy was sufficient for the first experiments, fluctuations in impedance and delivered energy did occur. The predefined energy ablation would solve this issue. As stated in the Introduction, one of the goals of this research was to develop a universal RFA platform. The device that we developed overcomes some issues that we encountered with commercially available instruments. We introduced a standard BNC connector to the generator to allow seamless integration of custom catheters. Another issue is the absence of protective mechanisms in the designed generator, that is, the impedance check in the ERBE instrument which caused difficulties when using the Habib EndoHPB catheter. Our generator is designed to accept any catheter design and deliver an AC signal with a specified voltage in a specified dose. Histological analyses revealed that required mucosal ablation was achieved. The thermal injury was limited to the epithelium and the lamina propria mucosae with sparing of the muscularis mucosae and deeper structures. Sham operation was performed to rule out possible artificial mechanical damage to the tissue caused by insertion and inflation of catheter that would cause unnecessary confusion by histological evaluation. Moreover, solely mechanical damage would not show thermocoagulative artifacts that we found after thermal injury. Samples harvested after sham operation showed no signs of tissue damage. The primary outcome of this project was feasibility and efficacy of the procedure and long-term survival was not thoroughly explored. Hence the risk of delayed complications, such as peritonitis, perforation of the intestinal wall, or pancreatitis, is unknown. Animals in our project, which were left to live 14 days after the procedure, showed no signs of the above-mentioned complications. In samples obtained 14 days after the procedure, there were no detectable morphological changes to the lamina propria mucosae. Given the verified histological changes in specimen harvested immediately after the procedure, the failure of intervention is not probable. A possible explanation for the absence of detectable structural changes 14 days after the procedure is reepithelialization of the ablated area. This option is to be further explored, as long-term tissue modifications induced by RFA may not necessarily be only structural but also functional (e.g., alteration in enteroendocrine cells' populations). This could present further potential application of thin-layer RFA in DMR, as duodenal mucosal resurfacing is also a procedure requiring superficial ablation, with subsequent evaluation of its possible impact on metabolic signaling. According to recent discoveries, the duodenum and its population of enteroendocrine cells responsible for the incretin effect play a significant regulatory role in glucose homeostasis. Observations in both animal and human studies reveal morphologic and functional changes in the proximal small intestine, such as abnormal mucosal hypertrophy, hyperplasia of enteroendocrine cells, and increase of enterocyte numbers in the presence of diabetes [27–29], implying a key role of the duodenum in the development of metabolic diseases including type 2 diabetes [30, 31]. Given these findings, a project assessing the efficacy of RFA as a method for DMR with the use of ZDF rats (Zucker diabetic fatty, an animal model for type 2 diabetes mellitus) was recently started. Besides its possible specific use in DMR, we further speculate about the additional application of our platform in various medical conditions. New approaches for the radiofrequency treatment of benign biliary strictures (BBS) are explored, some of them with promising results, especially for refractory cases [32]. However, available data on the use of RFA in this indication is still insufficient and is obtained from limited samples. Among the reported limitations of RFA in the case of BBS are the heterogeneity of the stricture etiologies and the diverse localization leading to difficult interpretation of the results. Furthermore, the distance between commonly used electrodes is too long (2,5 cm in Habib Endo HPB), which is usually longer than the stenotic part of the bile duct in BBS, and it could lead to unintended thermal injury [33]. We assume that an inflatable device capable of superficial ablation could find its utility in such cases. We estimate that, apart from gastroenterology, other medical fields could benefit from such devices. RFA can be used also in minimally invasive procedures in urology (e.g., in treatment of benign prostatic hyperplasia-BPH). The meta-analysis by Bouza et al. compared RFA versus transurethral resection of the prostate (TURP), showing that RFA-based methods significantly improved BPH parameters, although it does not reach the same long-lasting success as TURP. However, RFA seems to be an attractive option for patients with high anesthetic risks due to its safety, symptomatic alleviation, short duration of the procedure, and significantly lower number of complications than TURP, such as postprocedure bleeding, erectile dysfunction, incontinence rate, and stricture formation [34, 35]. We hypothesize that the construction of RFA balloon catheters could present another treatment option in candidates not suitable for resection methods or in early stages of symptomatic BPH, mostly due to its capacity to be inflated within the urethra, its presumed completely circular effect, precise depth, and continuous area of ablation. In pneumology, percutaneous RFA was introduced in inoperable patients with lung tumors with good results in the year 2000 [4]. In this method, the RFA electrode is placed under CT-imaging guidance directly into the tumor. During this procedure, complications such as pneumothorax, pleural effusion, or even hemothorax frequently occur. Moreover, this method lacks real-time treatment assessment and has limited access to central lesions due to the proximity of large vessels. To overcome these limitations, several transbronchial RFA devices have been developed and introduced into clinical use [5]. Most recently, a report by Motooka et al. described the feasibility of a prototype RFA device deployed from a standard endobronchial ultrasound bronchoscope (EBUS) in a preclinical animal study [7]. All these solutions consist of rigid needle-tip RFA electrodes. We assume that an inflatable RFA catheter inserted endobronchially would provide clinical benefit, especially in the central and mid-lung region by debulking of peribronchial lesions or airways obstructing lesions, particularly in poor candidates for surgery.

Our project was primarily exploratory. The primary goal was to test the technical feasibility of RFA with the use of our custom devices, optimizing the energies required to achieve the required biological effect (uniform and superficial tissue destruction). Small sample size may be perceived as a limitation. However, the statistical evaluation of the method's efficacy was not the primary outcome of our project. In the future, the utility and safety of our devices must be confirmed in further analyses.

## 6. Conclusions and Future Directions

In conclusion, RFA with the use of our prototype balloon catheter and generator optimized for low-impedance tissue in an animal model was feasible and safe to perform. Histopathological analyses confirmed successful superficial mucosal ablation with the preservation of deeper tissue layers. These are prototype devices and pilot experiments. Further improvements of hardware and software are needed to develop more predictable and repeatable results (one of the possible solutions would be direct printing of the conductive interdigitated array onto the balloon itself). This method of microendoluminal thin-layer ablation may represent a valuable treatment option in multiple benign and malignant conditions.

## Figures and Tables

**Figure 1:** Photomicrograph of rat small intestine without achieving targeted tissue destruction in pilot experiments (H&E). (a) With the use of Habib Endo HPB probe: small focal changes with thermocoagulation artifacts (hyperchromatic, elongated nuclei, and hypereosinophilic cytoplasm) limited to the upper part of villi surrounded by vital mucosa. (b) Our balloon-based catheter: vital mucosa of small intestine without detectable changes to epithelium.

**Figure 2:** Balloon-based bipolar RFA catheter—prototype.

**Figure 3:** Comparison of Habib EndoHPB catheter with the novel catheter: (a) circular but not laterally consistent ablation with EndoHPB catheter; (b) fully circular and laterally consistent ablation with the novel catheter using poultry liver in the ex vivo experiment.

**Figure 4:** RFA generator.

**Figure 5:** (a) Preparation of the operation field. (b) Insertion of RFA catheter. (c) Catheter inflated in proximal duodenum (white arrow). (d) Suture of the wound, end of the procedure.

**Figure 6:** (a) Endoscopic evaluation of RFA effect; (b) a direct endoluminal image of ablated mucosa (white arrow).

**Figure 7:** (a) Photomicrograph of rat nonablated proximal small intestine (H&E). (b) Rat proximal small intestine—acute effect of RFA—sample taken immediately after procedure showing ulceration with adjacent fibrin coagulum and intact lamina muscularis mucosae. (c) Rat proximal small intestine—subacute effect of RFA—24 hours after the procedure—transmural necrosis, a sharp transition area between ablated and nonablated mucosa (H&E). (d) Rat proximal small intestine—14 days after the procedure—no structural epithelial changes (H&E).

## Data Availability

The data are available upon request from the corresponding author.
